# A Novel Context Aware Joint Segmentation and Classification Framework for Glaucoma Detection

**DOI:** 10.1155/2021/2921737

**Published:** 2021-11-05

**Authors:** S. Sankar Ganesh, G. Kannayeram, Alagar Karthick, M. Muhibbullah

**Affiliations:** ^1^Department of Artificial Intelligence and Data Science, KPR Institute of Engineering and Technology, Coimbatore, 641407 Tamil Nadu, India; ^2^Department of Electrical and Electronics Engineering, National Engineering College, Kovilpatti, 628503 Tamil Nadu, India; ^3^Renewable Energy Lab, Department of Electrical and Electronics Engineering, KPR Institute of Engineering and Technology, Coimbatore, 641407 Tamil Nadu, India; ^4^Department of Electrical and Electronic Engineering, Bangladesh University, Dhaka 1207, Bangladesh

## Abstract

Glaucoma is a chronic ocular disease characterized by damage to the optic nerve resulting in progressive and irreversible visual loss. Early detection and timely clinical interventions are critical in improving glaucoma-related outcomes. As a typical and complicated ocular disease, glaucoma detection presents a unique challenge due to its insidious onset and high intra- and interpatient variabilities. Recent studies have demonstrated that robust glaucoma detection systems can be realized with deep learning approaches. The optic disc (OD) is the most commonly studied retinal structure for screening and diagnosing glaucoma. This paper proposes a novel context aware deep learning framework called GD-YNet, for OD segmentation and glaucoma detection. It leverages the potential of aggregated transformations and the simplicity of the YNet architecture in context aware OD segmentation and binary classification for glaucoma detection. Trained with the RIGA and RIMOne-V2 datasets, this model achieves glaucoma detection accuracies of 99.72%, 98.02%, 99.50%, and 99.41% with the ACRIMA, Drishti-gs, REFUGE, and RIMOne-V1 datasets. Further, the proposed model can be extended to a multiclass segmentation and classification model for glaucoma staging and severity assessment.

## 1. Introduction

Glaucoma is a common ocular disease caused by high intraocular pressure, which can eventually lead to irreversible blindness. It is a complex disease, influenced by patient's age, race, refractive error, OD, and retinal nerve fiber layer (RNFL) [1]. OD is an important indicator of glaucoma, where changes like cupping and thinning of RNFL are the most common signs of glaucoma. By exploiting the changes of OD, glaucoma can be detected in the early stages to prevent adverse outcomes. Different types of glaucoma have similar OD appearances and it is crucial to develop a framework for glaucoma detection that is robust to OD variability.

Several clinical studies have been performed to elucidate the relationship between glaucoma and the OD in terms of its structural changes, including thinning, cupping, excavation, and disc hemorrhage. One such investigation before two decades reported in [2] describes several OD variables and their ranking for early detection of glaucoma. Later, a systematic [3] approach for glaucoma detection defines five assessments of OD regions, viz., size of OD, shape, and area of rim, identification of RNFL loss, para papillary atrophy (PPA), and hemorrhages. In line with this, the significance of the examination of OD parameters in the differential diagnosis of glaucoma is presented in [4]. A most recent review [5] in this context brings out the risks of undiagnosis and overdiagnosis of glaucoma due to overlapping symptoms between glaucomatous and nonglaucomatous optic neuropathy in the OD region. Further, a recent case study also shows that constrictive ODs manifest in pediatric patients with central retinal vein occlusion (CRVO) [6], one of the important causes of glaucoma. These investigations show that the clinical importance of ODs in glaucoma detection is well recognized in ophthalmology research community.

Classification of glaucomatous disc changes is challenging due the mixed morphological manifestations of hemorrhage patterns on the surface of the OD. Cup to disc ratio (CDR) [2], evaluated as the ratio of vertical cup diameter (VCD) to vertical disc diameter (VDD), is one of the common measures for detecting glaucoma. A larger CDR signifies a higher risk of glaucoma. However, VCD is subjective, and the estimation of the OD's shape from fundus images, especially from the images taken through the OD's boundary, is also difficult. It is also challenging to find out the location of the OD's boundary for detecting cup shapes, especially when the eye is rotated to image the OD. CDR is evaluated by segmenting the OD and optic cup (OC) regions and computing the VCD to VDD ratio. The earlier approaches for automated glaucoma screening are called measurement-based approaches [7–10] which segment the ODs and cups followed by CDR computation.

Segmentation of ODs and cups is a nontrivial problem where inaccurate segmentations may result in false detections. In the recent years, deep learning approaches are gaining popularity in the deployment of automated glaucoma detection. Deep learning networks capable of learning image features at various levels of abstraction are employed as feature extractors and classification and segmentation models in glaucoma screening. Several two-stage convolutional neural network- (CNN-) based glaucoma detection frameworks which perform segmentation followed by classification are proposed in [11–14]. In the recent years, there is an increased attention on deep learning models for joint segmentation [15] of ODs and OCs which are rather complex to implement. However, these approaches are demonstrated to achieve superior performances compared to the conventional OD and OC segmentation based glaucoma detection models.

Existing works in literature pay less attention to the contextual information in glaucoma screening. While the models which segment the OD and OC separately focus on clear separation of boundaries for CDR calculation, the joint segmentation approaches are based on heavy learning models such as generative adversarial networks (GAN) and ensemble-based architectures. This research presents a context aware joint segmentation and classification framework for glaucoma detection based on the aggregated transformations and class activation maps (CAM). The framework called GD-YNet follows a YNet architecture [16] comprising a segmentation subnetwork and a classification branch. The segmentation subnetwork is trained on the region of interest (RoI) images encompassing the OD, captured from contextual features of activation maps to segment the ODs. The classification branch is constructed with a convolutional layer and two fully connected layers, and it is trained with a combination of low-level image features and the segmented disks and for binary classification.

The contributions of this research are as below.

1. A joint segmentation classification framework based on Ynet architecture which demonstrates superior OD segmentation and glaucoma classification performances is proposed
2. A hierarchical approach for RoI segmentation based on class activation maps (CAM) and aggregated transformations is proposed
3. The prosed framework is designed to harnesses the low-level and structural features of the fundus image in glaucoma detection

The proposed joint model is trained and tested with public databases, demonstrating superior segmentation and classification performances. From the objective metrics and explainable analysis, it is seen that the proposed model is a prospective solution for integration with glaucoma screening pipelines for better clinical outcomes.

Rest of this paper is organized as below. In Section 2, representative works on deep learning-based glaucoma detection models are reviewed.  Section 3 presents the datasets and underlying methods employed in building the proposed system. In Section 4, the architecture of the proposed model and subnetworks is presented with the training mechanism. Experimental results and their interpretations are presented in Section 5, and the paper is concluded in Section 6.

## 2. Related Works

Existing deep learning approaches for glaucoma detection are based on feature extraction, object recognition, transfer learning, RoI segmentation, OD and OC segmentation, and feature discrimination. The earliest deep learning model for glaucoma detection proposed in [17] is deployed as a six layered CNN with four convolutional and two fully connected layers. This model is trained on the augmented ORIGA [18] dataset and tested with the ORIGA and SCES [19] datasets achieving area under curve (AUC) values of 0.831 and 0.887, respectively. Realizing the significance of context information, the authors of [17] have proposed Automatic feature Learning for glAucoma Detection based on Deep LearnINg (ALADDIN) [20], following a contextual training strategy which enables the model to adaptively learn deep features discriminating normal and glaucomatous images.

Later, several deep learning models for glaucoma detection based on OD and OC segmentation have been proposed. In [21], the conventional UNet [22] which follows an encoder-decoder architecture is modified with dropout regularization, reducing the number of filters for OC and OD segmentation, achieving improved segmentation accuracies compared to conventional approaches. An ensemble learning-based CNN proposed in [23] employs entropy sampling to select highly informative points to reduce computational overheads. Further, it follows a gentle Adaboost approach for learning the filters in each convolutional layer. RACE-Net [24] based on a recurrent neural network models a generalized level set-based deformable model (LDM) to capture high-level dependencies between points on the object boundaries. It iteratively segments the ODs and OCs from a RoI, learning curve evolution velocities in each time-step, in an end-to-end manner. A multitask CNN [25] for joint segmentation of OD and OC and glaucoma detection is implemented by adding a classification branch to the classic UNet. The UNet is trained to jointly segment the OD and OC from the rough RoI segmented from the fundus image by intensity thresholding. The appearance features extracted at the encoder path are concatenated with the segmentation maps generated by the decoder path and a feature vector is constructed by global average pooling. A fully connected layer with a single neuron detects the presence of glaucoma from this feature vector. This model trained and tested with the REFUGE [26] dataset achieves a dice coefficient (DC) of 0.96 for OD segmentation and a sensitivity of 0.88 and a specificity of 0.91 for glaucoma detection.

A dual machine learning system [27] is built with two UNets, one each for disk and cup segmentation and a MobileNetV2-based classifier [28]. Features extracted from the localized disk and cup regions are used to evaluate the CDR, and the classifier is trained to detect glaucoma with the entire fundus image. Finally, a reporting tool is used to present the parameters such as adequacy of the size and shape of the segmented disk and cup, CDR, images of the segmented disk and cup, and classification score to an ophthalmologist. This system reports a classification accuracy of 86% on the Drishti-gs dataset [29] with the MobileNetV2-based classifier. However, the significance of the discreteness of the subsystems and nondependency between segmentation results and classification has not been justified by the authors.

In [15], OD and OC joint segmentation is modeled as a multilabel segmentation problem. A one stage network called the M-Net is implemented with an encoder-decoder architecture similar to UNet, extended with multiscale input and a side-output layers. Initially, disk center of a fundus image is localized by a deformable model, and the fundus image is transformed into polar coordinates. The multiscale pyramid of this image is fed as input to the input layer, and segmentation maps are constructed at the side-output layers. Finally, these maps are fused, and an inverse polar transformation provides the segmentation mask. This network achieves best segmentation results on the ORIGA dataset and superior classification accuracies with ORIGA and SCES datasets.

A depth guided semantic segmentation network is employed in [30] for joint segmentation of ODs and OCs. Initially, a fully connected convolutional network (FCN) with dilated residual inception blocks is trained to extract depth maps from the fundus images. Experimental results show that sparse fusion of depth information provides better segmentation results with small overlapping errors. Further, this framework is extended to glaucoma detection by thresholding the CDRs computed from the segmented ODs and OCs. The pseudodepth version of this model achieves an AUC of 0.8404 for glaucoma detection with the ORIGA dataset.

RetinaGAN [31] based on GAN for retinal vessel segmentation is extended to OD segmentation. This framework is implemented in four versions with a U-Net architecture as an encoder and four GANs such as Pixel GAN, Patch GAN-1, Patch GAN2, and Image GAN as decoders. Though this model demonstrates significant improvement in vessel segmentation, no such improvement is evidenced with OD segmentation.

The context encoder network CENet [32] captures high-level semantic information and preserves spatial information for semantic segmentation of medical images. It comprises feature encoder, context extractor, and feature decoder modules. The feature encoder employs a pretrained ResNet34 blocks for feature extraction. The context encoder is implemented with dense atrous convolution (DAC) and residual multikernel pooling (RMP) blocks to construct high-level semantic feature maps from these features, which are fed to the feature decoder modules to generate segmentation masks. This model reports small overlapping errors in OD segmentation compared to the classic UNet and other baseline models.

A spatial-aware neural network (SAN) [33] based on atrous CNN, pyramid filtering, and spatial-aware segmentation modules for joint OD and OC segmentation is a complex network which performs feature extraction in two stages. Initially, the local features are extracted with the Atrous CNN, and multiscale features are extracted from these feature maps with parallel pyramidal filters to construct spatial-aware feature maps. Segmentation is performed with spatial-aware segmentation blocks (SEB) which assigns class labels to the pixels by pixel-wise classification. This model is heavy due to the computation intensive architectural components.

A U-shaped CNN built with multiscale input and multikernel modules (MSMKU) proposed in [34] captures image features at multiple scales for improved segmentation. Further, this network is trained on Mixed Maximum Loss Minimization Learning strategy (MMLM) to train the network parameters, focusing on the samples exhibiting large training losses. Experimental results with RIMOne [35] and Drishti-gs datasets demonstrate superior performances with OD and OC segmentations and glaucoma detection.

In [36], joint segmentation of OD and OC is formulated as a semantic pixel-wise labeling problem. An encoder-decoder network called Cup Disc Encoder Decoder Network (CDED-Net) based on the fully connected SegNet [37] architecture is proposed, employing feature information reuse to bridge the semantic gap between the features shared between the encoder and decoder blocks. This model demonstrates state-of-the-art OD segmentation results with Drishti-gs, RIM-ONE, and REFUGE datasets.

Recurrent fully convolution network (RFC-Net) [38] is designed with recurrent units, multiscale input layer, and multiple output layer to capture high-level features of images and fine edges. Four types of recurrent units, each with a unique configuration of stacking the basic convolutional layers, are employed to evaluate the performance of the model for OD and cup segmentations. Experimental results show that best results are achieved with the stacked recurrent units achieving an accuracy of 0.9795 for joint segmentation of the disc and cup on the Drishti-gs dataset.

A disc-aware ensemble network (DENet) [39] is modeled as a binary classifier for glaucoma screening, guided by OD segmentation map. This network is implemented with four classification streams based on the fundus image, disc-cropped fundus image, disc segmentation map, and disc polar transform. The classification results from the four streams are combined by average ensembling to obtain a single classification score. This network achieves best AUC values of 0.9183 and 0.8173 on the SCES and SINDI [40] datasets, respectively, compared to conventional and deep learning based glaucoma screening models.

An adversarial learning framework called patch-based Output Space Adversarial Learning framework (pOSAL) [41] performs joint segmentation of ODs and OCs based on their morphologies. This network exploits unsupervised domain adaptation to minimize errors on segmentation with target datasets of diverse domains. In this framework, RoIs extracted from images of the source and target domains are fed as input to an adversarial segmentation network to predict the masks of the OD and OC. A discriminator follows the adversarial learning scheme to produce similar predictions for the source and unannotated target images. While segmentation loss is computed on the source images, adversarial loss is computed on the target images for generalization of the segmentation network. This network achieves a DC of 0.946 for the REFUGE validation dataset.

GLNet [42] is a multilabel segmentation model based on GAN for joint segmentation of ODs and OCs. The generator is a full convolutional network trained to construct the probability maps for OD and OC segmentation. The discriminator is implemented as an 8-layer network which assigns binary labels to the pixels, and it is optimized by minimizing the error between the predictions and the ground truth.

Though several deep learning frameworks are employed in OD and OC segmentation and glaucoma detection, exclusive studies to evaluate the performance of several deep learning classifiers on diverse datasets do not exist. One such investigation by Sreng et al. [43] presents a two-stage framework for OD segmentation in the first stage and classification of features extracted from the segmented ODs for glaucoma detection in the second stage. OD segmentation is performed using DeepLabv3+ [44] semantic segmentation network, employing ResNet18 [45], ResNet50 [45], XceptionNet [46], MobileNet, and InceptionResNet [47] as encoders. Performance evaluation of OD segmentation shows that best segmentation accuracy of 99.7% is achieved with MobileNet as the encoder of DeepLabv3+. Further, glaucoma detection is performed by employing three CNN based classification frameworks. The first framework employs pretrained CNNs for glaucoma detection by transfer learning, the second approach employs pretrained CNNs as feature extractors and trains SVM classifiers for glaucoma detection, and the third method creates an ensemble network of these two approaches. Each framework is evaluated with eleven CNNs, and the best glaucoma detection accuracy of 99.53% is achieved for the REFUGE dataset by the second framework with a pretrained DenseNet model [48] as a feature extractor.

The DenseNet supports feature propagation between layers with direct connections and facilitates feature reuse. The Fully Connected DenseNet (FC-DenseNet) model [49] for simultaneous OD and OC segmentation follows a U-shaped architecture. Glaucoma detection is performed by evaluating the CDR along the vertical and horizontal axes from the boundaries of the segmented ODs and OCs. In this approach, during preprocessing, the area within 2 optic disc diameter (2ODD) in the OD is cropped as the RoI for training the model. However, the mechanism for disk localization for cropping has not been revealed by the authors.

Despite several deep learning models deployed in glaucoma detection, surprisingly, new models following different learning paradigms have been proposed in 2020. A framework proposed in [50] for OD segmentation employs several basic machine learning operations such as binary masking, morphological opening, and estimation of the center of RoI for OD localization and cropping. From the cropped image, the highest peak value of the intensity is obtained with the improved Circular Hough Transform (CHT) to define the boundary of the OD. The circular region of the image captured around the peak is further subjected to superpixel segmentation in the red channel to segment the OD. Though this discrete framework reports a segmentation accuracy of more than 99% for different datasets, it does not provide a classifier model, learning features from these datasets for testing new images acquired.

The fuzzy broad learning system (FBLS) [51] for glaucoma screening employs two flat broad networks with fuzzy reasoning abilities for OD and OC segmentation. In this system, the RoI is extracted from the fundus image by directional matched filtering and level set segmentation, and the red and green channel images of the RoI are given as input to the OD and OC segmenting flat broad networks, respectively. Glaucoma detection is performed by computing the CDR from the segmented ODs and OCs. The authors report that optimal results are achieved with preprocessing and postprocessing the images. However, the postprocessing mechanism is not explicitly described.

Three representative deep learning models for glaucoma detection are proposed in 2021, each following an unique architecture. A two-stage glaucoma detection model proposed in [52] employs pretrained AlexNet [53], InceptionV3, InceptionResNetV2, and NasNet-Large [54] models in the first stage for glaucoma prediction, and these predictions are combined in the second stage by an ensemble classifier. Two approaches, namely, accuracy-based weighted voting and accuracy/score-based weighted averaging are used in ensembling the predictions of the discrete classifiers. Experimental results show that NasNet-Large demonstrates superior glaucoma detection accuracy of 99.3%, averaged on five different datasets. Further, accuracy/score-based weighted ensembling improves the average detection accuracy to 99.5%.

An attention UNet [55] constructed by adding an attention gate (AG) to the conventional UNet is fine-tuned with the DRIONS-DB and Drishti-GS datasets for OD and OC segmentation. Experimental results show a noticeable improvement in performance metrics of the model under transfer learning, with a smaller training dataset.

A convolutional autoencoder- (CAE-) based segmentation network for OD segmentation is proposed in [56]. Initially, the CAE is trained to learn the significant features from unlabeled fundus images by unsupervised learning, and it is transformed into a segmentation network by adding a convolutional layer with a 3 × 3 filter after the final convolutional layer of the decoder blocks of the CAE. This network learns to segment an OD, from an annotated set of fundus images. The convolutional layer employs a sigmoid activation function to construct the binary mask of the segmented OD.

From a thorough review of automated glaucoma detection literature, it is evident that context aware segmentation approaches yield best classification results in glaucoma screening, rather than conventional classifiers based on extraction of deep features from the fundus images. Recently, joint segmentation methods are getting wide research attention due to the simplicity of the design. However, their implementation is complex due to the intricacies involved in deploying them as multilabel segmentation approaches. Further, there are few works on multitask learning such as [16, 25] which combine segmentation and classification in a unified YNet framework. These models are realized by adding a classification branch to the segmentation networks. It is seen that this framework is promising as it considerably reduces the number of network parameters.

## 3. Materials and Methods

This section presents the training and testing datasets employed in this research and a succinct description of the underlying methods.

### 3.1. Datasets and Implementation Details

The public datasets, viz., ACRIMA, Drishti-gs, REFUGE, RIGA, and RIM-ONE are employed in training and testing the proposed system. The unified segmentation and classification model proposed in this research is trained and tested with discrete datasets without any data augmentation, to evaluate its generalization ability. The details of the datasets are given in Table 1.

The proposed framework is implemented with Matlab 2021a software, employing the image processing and deep learning toolboxes. The model is trained and tested with a NVIDIA GeForce GTX1060 3GB Graphics card enabled i7-7700 K processor with 32GB DDR4 RAM.

### 3.2. ResNeXt Architecture

Training deep networks is challenging due to the vanishing gradient and gradient explosion issues. To solve these problems, the residual learning approach was proposed in [45]. In this method, each layer in a deep neural network is equipped with a skip connection, and each layer of residual block is designed to learn the residual of the last layer and the layer itself. Therefore, the gradient of the activation of each layer can be propagated through the whole network to avoid the gradient vanishing or exploding. To obtain higher accuracy, the convolutional layers in the residual block are followed by the global average pooling (GAP).

The ResNeXt architecture [57] is an extension of the ResNet which replaces the standard residual block with a ResNeXt block which leverages a split-transform-merge strategy for aggregated transformations. In the ResNeXt architecture, the original input is split into a series of residual branches, each of which is followed by a series of point-wise convolutions and an element-wise sum. The output of the last layer of the network is then concatenated with the input to produce the output of the network. This architecture introduces a new parameter called cardinality, i.e., the size of the group of transformations which is demonstrated to improve classification accuracy. The schematics of the residual and ResNext blocks are shown in Figure 1. This architecture is leveraged with the layered CAM in the localization of the RoI in the proposed system.

### 3.3. Layer CAM

The CAMs generated from the final convolutional layer of a CNN provide a visual representation of the behavior of the classifier model, highlighting the areas of the image which are the most important for the classification. These maps are generated by first pooling the features of the neurons in the last layer of the CNN and then passing this information through a softmax function, to produce a probability distribution over the classes of the image. In this way, the activations of the final layer of the CNN can be viewed as a feature map, which can be interpreted as a visual representation of the model's classification decision, highlighting the topological and spatial distribution of its decision boundaries. The activation maps can be used in debugging the model to generate class-specific features for training a classifier.

However, CAMs are limited to classification problems, and using these coarse maps for localization is still a challenge. Jiang et al. [58] proposed an approach for fine-grained CAM construction exploiting the relationship between image gradients and feature maps. This approach generates a LayerCAM for fine-grained object localization, fusing the CAMs from the shallow and final convolutional layers. These hierarchical object locations can be interpreted from the corresponding gradient maps, which is important for understanding the role of each convolutional feature map.

In this research, the LayerCAM is constructed from the image gradients as described below. The weight of a spatial location (*i*, *j*) in a feature map *f* in a layer *l* is given in Equation (1) where *A*(∙) is the activation function.

(1) $$\begin{array}{c} W_{\left(i,j\right)}=A\left(g_{ij}^{f}\right) \end{array}$$

The activation of the entire feature map *f* is obtained by multiplying the feature values F_(*i*, *j*)_^*f*^and corresponding weights as in Equation (2). The LayerCAM is obtained as a linear combination of the activations of the feature maps as in (3).

(2) $$\begin{array}{c} \begin{array}{c} {\text{F}}_{\left(i,j\right)}^{\prime }={\text{W}}_{\left(i,j\right)}^{f}\times {\text{F}}_{\left(i,j\right)}^{f} \end{array}, \end{array}$$

(3) $$\begin{array}{c} C=A\left(\underset{f}{\sum }{\text{F}}_{\left(i,j\right)}^{\prime }\right). \end{array}$$

The schematic of LayerCAM construction is shown in Figure 2.

### 3.4. YNet Architecture

The proposed joint segmentation and classification model for OD segmentation and glaucoma detection is realized with a YNet architecture originally proposed in [16]. YNet facilitates convolutional modularity for generation of discrimination maps and class scores, along with segmentation, adding a classification branch to the basic UNet architecture. The UNet follows an encoder-decoder architecture with a contracting path and a symmetrical expansion path. The contracting path is a downsampling path, and the expansion path is a upsampling path. The encoding network learns to map an input image to a corresponding semantic map. It consists of a series of convolutional layers that progressively extract features from the input. These features are then upsampled to the original image resolution using transposed convolutions. The decoding network uses a mirror-like strategy to upsample the encoded image to the resolution of the input. It uses the upsampled features from the encoding network to predict the segmentation mask. Classification is performed from the features extracted at the lowest encoder layer of the UNet. The schematic of the basic YNet architecture is shown in Figure 3. This figure illustrates a clear separation of the UNet and YNet.

Generally, vanilla CNNs such as EfficientNet, Inception, ResNet, and VGG are employed as the backbones of the encoders and decoders defining the organization of the layers in the network. CNNs for image processing problems use fixed sized filters and exercising the networks to find optimal filter sizes requires an intensive tuning procedure, that is not easy to automate. Further, fixed size filters are suitable only for images with similar size salient parts, and they fail to adapt to images with varying scale. Inception networks employ filters of multiple sizes and shapes together in a single network. Such networks are shallow but can operate in a wide range of scales. The inception network is a deep convolution neural network that can be trained to detect salient regions in any image, and it can be used to generate new images that contain the same salient elements. Inception networks contain layers with multiple sized and shaped filters. For each layer, a region-of-interest (ROI) is extracted, and a convolution is computed on the input image with the filters that are applied to the ROI. The results of these computations are concatenated with the results from the previous layer. This facilitates the network to learn to identify features of different sizes. In this research, YNet is constructed from UNet which is built on the Inception blocks. The structure of the inception block is illustrated in Figure 4 which shows filters of different sizes in each layer.

## 4. Proposed System

OD morphology is a powerful predictor of the outcome of medical and surgical treatment and is one of the most significant prognostic factors in the management of patients with chronic glaucoma. Heterogeneity of OD provides insight into the pathophysiology of glaucoma and is associated with disease progression. The proposed framework is realized in two stages, viz., RoI segmentation followed by joint OD segmentation and glaucoma detection as shown in Figure 5.

RoI segmentation is realized by constructing the LayerCAM from the feature maps of the ResNext subnetwork. Segmentation of OD and glaucoma detection is performed with the joint segmentation and classification subnetwork, implemented with the inception YNet network, unifying inception blocks and the YNet architecture described in the previous section. The schematic of this subnetwork is shown in Figure 6.

The basic Ynet proposed in [16] is only employed as the backbone of the proposed architecture. Each convolutional layer in the YNet is replaced by the inception module shown in Figure 4. The inception module includes multiple 1 × 1 convolutions, 3 × 3 convolutions, 3 × 3 max pooling, and cascaded 3 × 3 convolutions. Along the contracting path, the number of filters is doubled in each layer, and the height and widths of the feature maps are reduced by half. The inception module in each stage generates four feature maps from the input and concatenates them. It results in increase in depth of the feature map in each layer by 4. The feature maps are downsampled by maxpooling in each layer, which results in their width and height being halved in each layer until the center of the UNet is reached.

At the lowest layer of the network, the feature map from the encoder path is subjected to a set of four convolutions and shared with the inception module in the decoder path. The resulting feature map is upsampled, doubling the width and height and concatenated with the feature map generated in the encoding path at the same layer. This results in a subsequent increase in depth of the feature maps by 8. Finally, the feature map generated at the top most layer of the decoder path matches the dimensions of the input image, and it is convolved with a set of 1 × 1 convolutions, by which the depth of the feature map is reduced to match the number of class labels. A binary segmentation mask is constructed from this feature map applying a pixel-wise activation function. The OD is obtained by masking it with the fundus image, and it is downsampled by average pooling. The low-level feature map from the last encoder stage is upsampled to match the size of the OD and concatenated with it. The resultant image of size 256 × 256 is fed as input to a convolutional layer with two 3 × 3 filter to construct a feature map of size 128 × 128. This is followed by two fully connected layers with sigmoid activation functions. The first fully connected layer generates a feature vector of size 64 × 1, and the second one generates the class scores.

The inception modules consists of 1 × 1, 3 × 3, and 5 × 5 convolutional filters and max pooling layers, generating four feature maps from the input and concatenating them. The 3 × 3 and 5 × 5 filtering operations are preceded by 1 × 1 convolutions to reduce the number of channels, and the maxpooling layer is used to create an abstract representation of the feature map before 1 × 1 convolution. The inception module is designed on the premise that salient parts of medical images are of arbitrary sizes and are often localized in a small spatial region. Further, the features should be invariant under changes in the input size to maintain invariance between different scales of objects. The Inception modules with different filter sizes integrated with the UNet architecture can capture multiple scales of optic disc features with various orientations, which can be learned efficiently to discern the OD. It is to be noted that the size of the input image, the number of classes, and the number of inception modules are all parameters of the proposed framework. Further, training this network with the cropped or resized candidate RoIs extracted from the Layer CAMs can further simplify the segmentation process.

### 4.1. Experimental Setup and Model Training

The proposed system constitutes subnetworks for RoI segmentation, OD segmentation, and classification. The training parameters of the framework are listed in Table 2.

For RoI segmentation, as seen in Figure 5, the ResNext101 subnetwork is not trained end-end as it is used to construct the LayerCAM from the feature maps of the ResNext blocks. This network is constructed with 4 layers, each with a ResNext block with cardinality 32. The weights of the ResNext pretrained with the ImageNet1K dataset are reused in the generating the feature maps from the fundus images for construction of the LayerCAMs. The ResNext and the inception YNet models are trained with an initial learning rate of 0.001, decaying the learning rate by a factor 2 after every 20 epochs, following stochastic gradient descent with momentum (SGDM) optimization. A momentum of 0.9 ensures that the models are trained with significant contributions from the previous updates.

The objective function of the joint segmentation and classification framework is expressed as a combination of segmentation loss *L*seg and classification *L*cls as as described below. The network is optimized by alternating minimization of the segmentation loss and the classification loss in each iteration, thus improving the performance of both tasks. The objective function of the model is expressed in Equation (4).

(4) $$\begin{array}{c} \underset{\Theta ,y}{\min}\frac{1}{N}\overset{N}{\underset{i=1}{\sum }}\left[Lseg\left(F_{\theta }\left(x_{i}\right),y_{i}\right)+Lcls\left(y_{i}\right)\right]. \end{array}$$

In this formulation, *N* is the training set size, and *y*_*i*_ is the label of the segmentation mask for the sample *i* . The segmentation loss can be formulated as in (5).

(5) $$\begin{array}{c} Lseg=\frac{1}{\sigma \times N}\overset{N}{\underset{i=1}{\sum }}\;\left[1-y_{i}\right]||y_{i}-F_{\theta }\left(x_{i}\right){||}_{2}, \end{array}$$

where 1 − *y*_*i*_ denotes the binary crossentropy loss with *y*_*i*_, *F*_*θ*_(*x*_*i*_) is the predicted segmentation mask, and *σ* is the loss weight in the range [0 1]. The classification loss can be formulated as in (6).

(6) $$\begin{array}{c} Lcls=-\left(1-y_{i}\right)\log\left(y_{i}\right). \end{array}$$

In this minimization problem, *L*seg penalizes the deviation from the ground truth segmentation mask, while *L*cls encourages the segmentation to be as close to one as possible. *y*_*i*_ can be 0 or 1 depending on the ground truth and network predictions.

## 5. Experimental Results and Discussions

### 5.1. Segmentation and Classification Results

This section presents the OD segmentation and glaucoma detection results on the datasets. Initially, the RoI is localized with the LayerCAM constructed from each training image to capture the candidate ODs. The activations at different channels of a convolutional layer, and the LayerCAM construction are shown in Figures 7 and 8, respectively. The LayerCAM is subjected to binary thresholding to construct a mask, and the segmented RoI is obtained by masking the fundus image. These illustrations present visual interpretation of the activations at multiple learnable layers.  Figure 8 shows that the RoI encompassing the OD is captured by the CAMs at increasing levels of clarity from the first layer to the fourth layer. It is seen that the LayerCAM clearly localizes the RoI encompassing the OD. The joint segmentation and classification model is trained with these RoIs from the training images to segment the ODs for glaucoma detection.

The proposed inception-based YNet framework is initially fine-tuned for segmentation with the MESSIDOR dataset, and it is tested with the RIMOne-V2 dataset. The segmentation results for a subset of images are shown in Figure 9 for visual analysis. It is seen that the RoIs are segmented precisely from the fundus images, and the ODs segmented from them match the ground truth binary masks.

The segmentation and classification performances are evaluated with the accuracy, sensitivity, specificity, precision, DC, Jaccard coefficient (JC), structure measure (SM), and enhance-alignment measure (EM) metrics. The ground truths required for these evaluations are provided with the RIMOne-V2 dataset.

Accuracy is a measure of the number of correct predictions out of the total number of samples, which is derived from the true positive (TP), true negative (TN), false positive (FP), and false negative (FN) values as in (7).

(7) $$\begin{array}{c} \text{Accuracy}=\frac{\left(\text{TP}+\text{TN}\right)}{\left(\text{TP}+\text{TN}+\text{FP}+\text{FN}\right)}. \end{array}$$

While sensitivity and specificity refer to the proportions of true positives and true negatives correctly identified, respectively, in OD segmentation problem, these metrics refer to the number of correctly identified pixels of the OD and the background, respectively, as in Equations (8) and (9).

(8) $$\begin{array}{c} \text{Sensitivity}=\frac{\text{TP}}{\left(\text{TP}+\text{FN}\right)}, \end{array}$$

(9) $$\begin{array}{c} \text{Specificity}=\frac{\text{TN}}{\left(\text{TN}+\text{FP}\right)}. \end{array}$$

Precision refers to the number of correctly identified samples of the total number of predicted positive samples as in Equation (10).

(10) $$\begin{array}{c} \text{Precision}=\frac{\text{TP}}{\left(\text{TP}+\text{FP}\right)}. \end{array}$$

The dice metric, a measure of the overlap between the prediction *P* and the ground truth *G*, is given in Equation (11).

(11) $$\begin{array}{c} Dice=\frac{2\left|P\cap G\right|}{\left|P\right|+\left|G\right|}. \end{array}$$

JC also called intersection-union (I-U) measures the similarity and difference between the prediction and the ground truth.

(12) $$\begin{array}{c} \text{JC}=\frac{\left|P\cap G\right|}{\left|P\cup G\right|}. \end{array}$$

The SM which evaluates the similarity between the segmented mask and the ground truth based on object and region awareness is given in Equation (13), where *S*_*o*_, *S*_*r*_, *α*, *S*_*p*_ and *G* refer to the object-aware similarity, region-aware similarity, trade-off between object and region awareness, predicted mask, and the ground truth, respectively, where *α* = 0.5 by default.

(13) $$\begin{array}{c} SM=\left(1-\alpha \right)\times S_{o}\left(S_{p},G\right)+\alpha \times S_{r}\left(S_{p},G\right). \end{array}$$

EM is a measure of the global and local similarity between binary maps of the segmented and ground truth masks as given in Equation (14), where *w* and *h* are the width and height of ground truth mask *G*, and *φ* is the enhanced alignment matrix.

(14) $$\begin{array}{c} {\text{EM}}_{\varphi }=\frac{1}{wh}\overset{w}{\underset{x}{\sum }}\overset{h}{\underset{y}{\sum }}\varphi \left(S_{p}x,y\right),\left.G\left(x,y\right)\right). \end{array}$$

Given a prediction *S*_*p*_, EM_*φ*_ is obtained from a binary mask, thresholding each pixel in the range [0 255]. The alignment matrix *φ* captures the similarities between the predicted mask and the ground truth at the pixel and image levels, from the global means. All these metrics range from 0 to 1 and evaluate to a value closer to 1 when the predicted segmentation masks are similar to the ground truth. Segmentation metrics for the Drishti-gs dataset is compared with that of state-of-the-art models in Table 3.

From Table 3, it is evident that the best segmentation results are achieved by the proposed model except specificity. This shows the prevalence of false positives in the segmented ODs, which can be eliminated by localizing them by morphological analysis. In continuation, the classification subnetwork, modeled as a binary classifier, is trained with the ODs segmented from the RIMOne-V2 dataset for glaucoma detection. The classification results are presented in Table 4 for the ACRIMA, Drishti-gs, REFUGE, and RIMOne-V1 dataset in Table 4. It is observed that the proposed model achieves best results for the ACRIMA dataset. The confusion matrices depicting the classification performances are shown in Figure 10.

The receiver operating characteristics (ROC) of the classifier model for the four datasets are shown in Figure 11. It is observed that the curves and optimal operating points are consistent for all the datasets.

Further, a comparison of the classification results with representative works is presented in Table 5. Comparison of performance metrics for the four datasets shows that the proposed framework is superior to the state-of-the-art approaches. Best classification accuracies of the proposed model are attributed to the RoI segmentation from the CAMs from multiple convolutional layers and perfect segmentation of the ODs. It is seen that compared to the pretrained classification networks such as the shuffleNet, squeezeNet, and other inception networks fine-tuned with the glaucoma detection, the proposed framework which shares features across segmentation and classification tasks demonstrates superior performance. Further, it is also observed that misclassifications are highly pronounced with the normal images which signify a high FP rate.

### 5.2. Explainable Artificial Intelligence Analysis

Recently, explainable artificial intelligence (XAI) has emerged as one of the key methodologies to enable trust, acceptance, and adoption of machine learning models in several domains. XAI complements the learning models by providing transparent explanations for the decisions based on the data. Generally, XAI is performed with CAMs and gradient CAMs constructed from the final learnable layer of a deep learning model. In this paper, the LayerCAM construction for RoI segmentation is based on multiple CAMs as described in Section 3.4. In this research, gradient-CAMs (GCAM) [59] are employed in analyzing the behavior of the binary classification process. This analysis is performed by capturing the GCAM of the convolutional layer in the classification branch of the GD-YNet. The GCAMs and the class scores are shown in Figure 12 for classification of normal and glaucomatous images in the Drishti-gs dataset.

It is observed that the class scores for the correct classifications are closer 1 while they are comparatively lower for misclassifications. It is seen the GCAM for the misclassified normal image is very small, and that of the glaucomatous image is not intact. The GCAMs show that the ODs are of diverse morphologies for normal and glaucomatous images. A detailed analysis of the CAMs can facilitate the definition of the OD morphologies in the staging and severity analysis of glaucoma.

### 5.3. Ablation Study

Experimental results reveal that the proposed model demonstrates superior performance with few misclassifications on all test datasets. This shows that the experimental setup is ideal for the glaucoma detection problem. In this scenario, it is unrealistic to study the performance of the model by increasing the depth of the YNet architecture. Since the classification accuracy depends on the segmentation of the ODs, it is appropriate to perform ablation study with the ResNeXt network used in LayerCAM construction.

As shown in Figure 5, the proposed segmentation classification framework employs four ResNeXt blocks for LayerCAM construction. Ablation study is performed by reducing the number blocks to three and evaluating the classification performances on the ACRIMA, Drishti-gs, REFUGE, and RIMOne-V1 datasets. The effect of this study on RoI segmentation is shown in Figure 13. LayerCAM1 is constructed from the CAMs of the first three layers, and LayerCAM2 is constructed from that of all the four layers. It is evident that reducing the number of CAMs results in a loss of finer details for localization of OD and accurate OD segmentation. The classification results obtained under the ablation study are given in Table 6, and it is seen that there is a performance degradation by 5% compared to that of the proposed GD-YNet, implemented with the segmentation subnetwork with four ResNeXt blocks reported in Table 4.

## 6. Discussion

The efficacy of the proposed glaucoma detection model is established with the experimental results, comparative analyses, and explainable studies. Further, XAI analysis shows that OD morphologies of arbitrary shapes and sizes are captured by the proposed model. Superior performance of the proposed framework is attributed to the context aware RoI segmentation using LayerCAM. The ResNeXt model, commonly used as a pretrained classifier or encoder backbone in semantic segmentation networks, is employed as a feature extractor in the construction of LayerCAM. Several existing models initially perform cropping for RoI or OD segmentation. However, several images in the dataset captured at different orientations do not have the ODs oriented to the image centers, and cropping them results in loss of the RoI. To the contrary, the proposed model localizes the RoIs from the LayerCAMs constructed from the ResNeXt blocks aggregating the finer and coarse details of the OD.

The proposed GD-YNet resembles the joint segmentation and classification architectures of [16, 25]. The multitask CNN proposed in [25] is exclusively meant for glaucoma detection with color fundus images. However, this framework requires a rough RoI segmentation based on intensity thresholding and Hough Transform. Further, it follows a complex postprocessing procedure to refine the segmentation results. Also, binary thresholding and morphological operations are performed on the segmented masks to separate the ODs and OCs. Further, ellipse fitting is performed to segment the OD. This framework is tested with only the REFUGE dataset, and the classification accuracy is smaller compared to the GD-YNet.

The Ynet proposed in [16] for joint segmentation and classification of breast biopsy images generalizes the conventional UNet with a classification branch. This network requires the RoI of the biopsy image to be fed into the YNet for further segmentation and classification. This network is implemented with residual convolutional blocks (RCB) and efficient spatial pyramid blocks (ESP) in the encoder and decoder paths. An increase in 4% accuracy is witnessed, increasing the depth of this network from 2 to 5.

Though the architecture of the proposed GD-YNet matches the schematic of the YNet, the proposed framework is superior to the works in [16, 25] in two main aspects. The proposed framework employs a context-aware RoI segmentation approach unlike the multitask CNN and YNet. Further, the encoder and decoder blocks of the GD-YNet are implemented with inception blocks, employing filters of varied sizes to capture features at multiple scales. While convolutional and deconvolutional filters are employed in multitask CNN, and the RCB and ESP blocks are employed in YNet, these architectures do not have the flexibility of the inception blocks used in the proposed GD-YNet. Inception networks offer several variants of the inception blocks with filter factorizations, towards label smoothing, improved optimization, and computational cost reduction.

In spite of the demonstrated efficacies of the proposed framework in segmentation and classification, certain limitations have been identified which must be addressed in future. The first limitation is concerned with the architecture of the ResNeXt blocks. The cardinality value of the ResNeXt blocks is arbitrarily assumed as 32. LayerCAM with different cardinalities and group convolutions can be used to study the performance of the model with respect to these parameters towards optimization of the cardinality and filter sizes. The second limitation is the usage of the basic inception modules with dimension reduction abilities in the encoder-decoder paths. Recently, variants of inception networks have been introduced with factorized 7 × 7 convolutions, root mean square (RMS) optimizers, and reduction blocks. The naïve inception blocks may be replaced by these variants for improved performances.

## 7. Conclusion and Future Directions

This paper presents a novel framework based on YNet architecture for joint segmentation and classification in glaucoma detection. It is implemented in two stages with context aware RoI segmentation, leveraging the potential of the aggregated transformations of the ResNeXt architecture in the first stage and a light-weight classification branch in the second stage. The proposed GD-YNet model based on this framework is trained to segment the ODs from the segmented RoIs followed by binary classification from the ODs. Tested with public datasets, this framework demonstrates superior segmentation and classification performances compared to state-of-the-art models. Chronic glaucoma manifests diverse morphological patterns in the ODs such as disc hemorrhage, nerve fiber layer defects, nerve fiber layer swelling, and atrophy. The proposed framework can be extended to multiclass segmentation and classification in the detection of pathologies pertaining to neuroretinal rim losses, disc cupping, rim thinning, disc hemorrhage, etc. This requires extensive training of the proposed model with several classes to differentiate morphological patterns of the ODs.

## Figures and Tables

**Figure 1:** Architecture of (a) residual block. (b) ResNext block.

**Figure 2:** Layer CAM construction.

**Figure 3:** YNet architecture.

**Figure 4:** Architecture of inception block.

**Figure 5:** Joint OD segmentation and glaucoma detection framework.

**Figure 6:** GD-YNet architecture with inception blocks in YNet.

**Figure 7:** Channel activations for a fundus image.

**Figure 8:** LayerCAM construction and OD segmentation.

**Figure 9:** Segmentation results for RIMOne-V2.

**Figure 10:** Confusion matrices for classification: (a) ACRIMA, (b) Drishti-gs, (c) REFUGE, and (d) RIM-One.

**Figure 11:** ROC for classification: (a) ACRIMA, (b) Drishti-gs, (c) REFUGE, and (d) RIM-One.

**Figure 12:** XIA on glaucoma detection.

**Figure 13:** Ablation study-LayerCAM construction and OD segmentation.

**Table 1:** Training and testing datasets.

Stage	Data set-no. of training images	Data set-no. of testing images
OD segmentation	RIGA-750	RIM-ONEv2-455

Glaucoma detection	RIM-ONEv2 Glaucomotous-200 Normal-255	ACRIMA Glaucomotous-396, normal-309 Drishti-gs Glaucomotous-70, normal-31 REFUGE Glaucomotous-40, normal-360 RIM-ONEv1 Glaucomotous-51, normal-118

**Table 2:** Training hyperparameters of GD-YNet.

Parameter	Values
Maximum epochs	100
MiniBatchSize	128
Momentum	0.9000
Learning rate	0.001
Optimization	SGDM
L2 regularization parameter	0.001
No. of paths (ResNext)	32
No. of ResNext blocks	4
No. of layers (YNet)	4

**Table 3:** Segmentation results comparison with state-of-the-art-Drishti-gs.

Model/method	Accuracy	DC	JC	Sensitivity	Specificity	SM	EM
Modified UNet [21] Sevastopolsky (2017)	—	0.9043	0.835	0.9156	0.9969	—	—
Ensemble CNN [23] Zilly et al. (2017)	—	0.973	0.914	—	—	—	—
RACE-Net [24] Chakravarty and Sivaswamy (2018)	**—**	0.97	**—**	**—**	**—**	**—**	**—**
M-Net [15] Fu et al. (2018)	**—**	0.9678	0.9386	0.9711	0.9991	**—**	**—**
FC-DenseNet [49] Al-Bander et al. (2018)	0.9969	0.949	0.9042	0.9268	0.9992	—	—
Retina- GAN (pixel GAN) [31] Son et al. (2019)	**—**	0.9674	**—**	**—**	**—**	**—**	**—**
SAN [33] Liu et al. (2019)	**—**	0.98	—	—	—	—	—
U-Shaped CNN with MSMKU [34] Xu et al. (2019)	**—**	0.9780	0.9496	0.9792	0.9994	**—**	**—**
Dual UNet+MobileNetV2 [27] Civit-Masot (2020)	—	0.93	—	—	—	—	—
CDED-Net [36] Tabassum et al. (2020)	**—**	0.9597	0.9183	0.9754	0.9973	**—**	**—**
RFC-Net [38] Gao et al. (2020)	0.9764	0.9787	—	0.9578	0.9783	—	—
Improved Image Processing Algorithms [50] Ramani and Shanthamalar (2020)	0.9922	0.8663	—	0.9495	0.9934	—	—
FBLS [51] Ali et al. (2020)	—	0.968	—	—	—	—	—
Attention UNet [55] Zhao e al. (2021)	0.9975	0.9638	0.9301	0.9488	0.9993	—	—
CAE [56] Bengani and Vadivel (2021)	0.9957	0.967	0.9314	0.9539	0.9993	—	—
GD-YNet (proposed)	0.9986	0.9945	0.9971	0.9812	0.9801	0.8271	0.8045

-Not reported.

**Table 4:** Classification results for four test datasets.

Dataset	Accuracy	Sensitivity	Specificity	Precision	FPR	F1	MCC
ACRIMA	0.9972	1	0.9935	0.9950	0.0065	0.9975	0.9943
Drishti-gs	0.9802	0.9857	0.9677	0.9857	0.0323	0.9857	0.9535
REFUGE	0.9950	1	0.9944	0.9524	0.0056	0.9756	0.9732
RIMOne-V1	0.9941	1	0.9915	0.9808	0.0085	0.9903	0.9861

**Table 5:** Classification results comparison with state-of-the-art for four test datasets.

Dataset	Model	Accuracy	Sensitivity	Specificity	AUC
ACRIMA	GD-YNet (proposed)	0.9972	1.0	0.9935	1.0
	XceptionNet [11] Diaz-Pinto et al. (2019)	0.7021	—	—	0.7678
	DenseNet [43] Sreng et al. (2020)	0.9953	—	—	0.9998
	AlexNet [52] Taj et al. (2021)	0.995	1.0	0.989	—
	InceptionV3 [52] Taj et al. (2021)	0.985	0.991	0.977	—
	InceptionResNetV2 [52] Taj et al.(2 021)	0.990	1.0	0.977	—
	NasNet-Large [52] Taj et al. (2021)	0.995	0.991	1.0	—

Drishti-gs	GD-YNet (proposed)	0.9802	1.0	0.9355	1.0
	OverFeat and VGG-S [12] Orlando et al. (2017)	—	—	—	0.7626
	XceptionNet [11] Diaz-Pinto et al. (2019)	0.7525	—	—	0.8041
	ShuffleNet [43] Sreng et al. (2020)	0.8667	—	—	0.7884

REFUGE	GD-YNet proposed	0.9950	1.0	0.9944	1.0
	Multitask CNN [25] Chakravartyand Sivswamy (2018)	—	0.88	0.91	0.96
	Ensemble +SVM [43] Sreng et al. (2020)	0.9575	—	—	0.9432

RIMOne-V1	GD-YNet proposed	0.9941	1.0	0.9915	1.0
	AlexNet [52] Taj et al. (2021)	0.875	0.836	0.904	—
	InceptionV3 [52] Taj et al. (2021)	0.922	0.891	0.945	—
	InceptionResNetV2 [52] Taj et al. (2021)	0.906	0.855	0.945	—
	NasNet-Large [52] Taj et al. (2021)	0.945	0.927	0.959	—
	VGG19 [14] Gómez-Valverde et al. (2019)	—	0.8701	0.8901	0.94
	XceptionNet [11] Diaz-Pinto et al. (2019)	0.7121	—	—	0.8575
	SqueezeNet [43] Sreng et al. (2020)	0.9737	—	—	1.0

-Not reported.

**Table 6:** Classification results under ablation study (No. of ResNeXt blocks is reduced to 3 from 4).

Dataset	Accuracy	Sensitivity	Specificity	Precision	FPR	F1	MCC
ACRIMA	0.9453	0.9516	0.9418	0.9433	0.0582	0.9486	0.9456
rishti-gs	0.9292	0.9344	0.9174	0.9344	0.0826	0.9374	0.9068
REFUGE	0.9433	0.9480	0.9427	0.9029	0.0573	0.9278	0.9255
RIMOne-V1	0.9424	0.9476	0.9399	0.9298	0.0601	0.9418	0.9378

## Data Availability

The data used to support the findings of this study are included within the article.
